RETRACTED

# Active Treatment of Water Chemistry for Swimming Pools Using Novel Automated System (NAS)

**DOI:** 10.1155/2022/5210225

**Published:** 2022-05-17

**Authors:** Saeed Asiri

**Affiliations:** Mechanical Engineering Department, Faculty of Engineering, King Abdulaziz University, Jeddah, Saudi Arabia

## Abstract

The Novel Automated System (NAS) has the control system of the level of chlorine and acid (i.e., pH level) through a feedback in three forms of synchronous alerts. The feedback is in the form of an alert voice, a visible color, and a message on a digital screen. In addition, NAS contains a slide-in container in which chemicals are used to treat the problems of chlorine and acid levels independently. Moreover, NAS has a net in front of it to clean the pool on the surface of the water from leaves and wastes and so on which is controlled through a remote control. The material used is a lightweight aluminum with mechanical and electric parts integrated with each other. In fact, NAS is qualified to serve as an assistant security guard for swimming pools because it has the characteristics that make it unique and smart.

## 1. Introduction

Swimming pool problems depend on the source of the problem either from human, climate, and environment conditions [1]. Many problems can happen for the swimming pool such as: chlorine reduction, pH decreases by time, and recreational water illnesses (RWIs) [2]. Following by, in 2001 a water park in the United States, around 360 people have gotten sick who contracted diarrhea, although there was an adequate level of chlorine and pH in the water [3]. In 1998 in Georgia, USA, 26 people showed symptoms of illness after swimming in a pool with a child who had Escherichia coli (see Figure 1) [4].

As a result, seven of the people were taken to hospital, but fortunately, the outbreak did not happen. Even, the chlorine levels were still same in the normal level. Subsequently, taking care of swimming pool problems gave awareness on how to avoid risks and make preventive measures [5]. Furthermore, NAS is very useful because it treats a real-life problem faced by many people using swimming pools.

A study says that people who are using chlorine for house cleaning have a less chance of being subjected to the risk of asthma, allergens, and microbial agents such as antitoxins [6–8]. Chlorine is used in wide range in local and international applications of swimming pools. It could be used for filtering swimming pools from bacteria that are caused by swimming action. In addition, it is useful for producing chemical and polymers objectives [9–12].

Filtering swimming pools is very important to stop microorganisms from growing. Swimming pool water contains higher amount of chlorine that has the capability of keeping the temperature of water consistently warm [8]. In a study on swimming pool safety and drowning risks, a number of 600 people with ages ranging from five to 24 years have died due to drowning in a period of two years [9]. As a result, on evaluation, it was because of the effect of containing the normal amount of acid to kill small size of bacteria in swimming pools that chlorine cannot kill them [10].

RETRACTED

Swimming pools are getting very popular inside of houses so that means the traditional way to take care of children away from falling in is very important. No doubt that using robots and technology life is being easier and better as well as cleaning swimming pools in traditional way is taking so much of time, effort, and money, so using smart boat to deal with this kind of cases is highly recommended [11].

Regarding the basic concepts of the control system of the smart boat especially in the chlorination treatment, Manzanilla [12–15] studied the nonlinear model of underwater robot at the UMI laboratory. The robot is composed of four rotors that produce forces and torques to move and stabilize it. The results were only on four degree of freedom and four control inputs, the body frame, buoyancy force, the angle, and the external forces. They did several simulations to prove the well performance of the closed loop.

Khattak et al. [13] have studied the underwater remotely operated vehicles in nonlinearity dynamics using simulation of MATLAB and Simulink in addition to the experiments to check the validation of the model. They also investigated the functional requirements of the ROV, which are the automatic movement and depth while it remote controlled. Papadopoulou [13] investigated the amount of the chlorine and pH acid in five different public swimming pools (three were indoors and two outdoors) in NW of Greece. The range sizes of the swimming pools were from 18 m^2^ (domestic pool) to 1250 m^2^ (competition pool), for the indoor pools to provide the Greek standard ranges for pH 7.2–7.8 and maximum free chlorine 2.5 mg/l with an automatic backwashing twice a week.

Asiri [14] has designed one or more processing units for powering the processing units along with two or more distance sensors, a power supply, one or more cells, and the motors from energy supplied by the solar cells. The processing units might be configured by one or more processing modules for planning and executing a traversal path across the water body surface. The signals were considered to establish a portion of the traversal path from distance sensors. The study contribution is a boat that provides innovative solution to adjust the level of chlorine and acid in the water. The design of a slider-crank mechanism, with gates which are containing the chlorine and acid medicine to be added to the swimming pool water if the sensor senses it is below the normal level. This boat also works as a life guard if any, child drown, by default he/she makes high motion, and so the boat feels that motion by a passive vibration sensor which sends an emergency signal to the remote control to produce a very loud alarm.

RETRACTED

## 2. Methodology

A state of art smart device shown in Figure 2 was invented in Mar.30, 2017 [15–17]. The device is connected to other devices via Internet and has the ability to monitor the pool as it is provided with an alert system. The device uses a buoy that can float inside the swimming pool water. Fundamentally, the device contains several sensors in which they work as measuring tools for different parameters that can provide the operation with a full awareness of the pool. The sensing devices can measure many data such as water pH level, water temperature, water salinity, level of pool water, ultraviolet (UV), and ORP indexes in water.

After the sensing devices read the measured data of a parameter, the data are transmitted via radio signals to the gateway where it analyzes and stores the data. The gateway stores the data in cloud servers. Therefore, it makes that data accessible to other different smart devices like phones, laptops, and PCs. The device also works as an alert system where it can alert and notify the operator to the variance of the measured data compared to the standard safety data that were set for pool safety. One of the most helpful sensing and alert features is that the device can alert the operator if a body or a person enters the pool water by measuring the water movement and its characteristics which can provide well safety to pool users/owners.

Figures 3 and 4 show that, on 17^th^ of May 2005, a smart flying boat has been created, and this smart boat is flying over the water by using a propeller. It consists of the main body, propeller, and two wings, while the wings connected to flaps one in the front and the other is in the back. That flap will be controlled by lifting the wings up and down. The propeller is placed at the lowest point of the boat which is connected to a vertical motor. There is a navigation system in the smart flying boat which consists of steering wheel, accelerate pedal, switches to control by engine movement, switches to control by flap movement also, and finally electrical circuit that is controlled by the motor and switches [16]. In addition, motion sensor has published in 11 Mar 1997. Logically, the motion sensor works by detecting motion of movement in general. It detects motion and converts them into electric-mechanical signals or by far read them by the favorite language which is electrical signals. After that, the sensor [17] provides the oscillator interruption to active signals.

RETRACTED

Hence, interruption once gives continuous series of the signal at a time. Somehow, condition alarm meets its satisfaction while interruption signals are detected through windows. The sensor contains conductive sphere within a cylinder to locate the sphere within conductive plates and internal surfaces. After that, internal surfaces are being followed to get the sphere to rest condition contacting the last surface of the sensor. To provide visible alarms, since the device detecting motion including jumper circuits which are small wire uses to connect elements through passing others inside the electric circuit so the jumper circuits are providing to the circuit casual motion as well as visible alarms. In addition, the next step is controlling through remote the sending and receiving signals which are converting later into alarms [18–20]. Excessive amount of chlorine in swimming pool water had caused symptoms of respiratory disease [14]. The symptoms have appeared in adults at a percent of 66.7% while for children it was 71.6%. For people who are experiencing respiratory diseases, the symptoms lasted a longer time compared to the other people [19–21].

Inspired by this project is the need to remotely control and monitor our children's pool, which is an Intex 15 'x 48 circular pool. The pool holds approximately 5000 litres of water. It is connected to a sand filter/pump, 11 kW heater, and saltwater system. The goal is to monitor the temperature of the pool water, air temperature and control the pumps, heaters, and salt water system to ensure that the pool is warm enough for the children without being overheated. Raspberry Pi, Arduino, IoT power supplies, and breadboards are attached to plastic storage containers with zippers to prevent water/moisture from entering boreholes for cables and ventilation.

A pair of DS18B20 waterproof temperature sensors is used to monitor the water temperature and air temperature of the pool. These sensors are connected to the Arduino Uno R3 through the Dallas Management Library and the OneWire Library. The temperature data (in degrees Celsius) is sent to the Raspberry Pi via I2C every 1 second. The two temperature values are separated by “|.” Some cheap speaker cords (doorbell cables) were used to extend the range of the DS18B20 which reads the water temperature. This DS18B20 was submerged in the pool.

(1) $$\begin{array}{c} \text{temperatureData}=\text{padRight}\left(\text{String}\left(\text{poolSensor}.\text{getTempCByIndex}\left(0\right)\right)+“|”+\text{String}\left(\text{outsideSensor}.\text{getTempCByIndex}\left(0\right)\right),L2C\text{ BUFFER LEN}\right). \end{array}$$

Figures 5 and 6 show the Raspberry Pi controls IoT power supply and connects the pump and salt water system to the 110 V power supply. This is done using a 3 V pin on the Pi. Replace the 3 V pin to turn 110 V connectors on/off the IoT power supply (the plug-in pairs are closed by default).

RETRACTED

## 3. Results

Figure 7 shows the overall view or isometric view of NAS. It characterized in offering three sensors for safety and filtering swimming pool water. As showing above, the vibration sensor is mounted on the top of the boat, the reason behind that is to give much more accurate readings in general. Chlorine and PH sensor are fixed in the front of the boat for keeping them away from boundaries of the boat as much as possible.

The sliders are mounted in the right and the left sides of the boat, which are containing chemical medicine when needed. Also, the fountain is designed in the front to give beauty for the boat and for the swimming pool itself. For a boat to float, it needs to weigh less than the same amount, or volume, of water. To make this happen, the boats must be built so that they have giant pockets of air inside them.

### 3.1. Buoyancy Force

Moreover, to calculate the buoyancy force [13], double half of boat weight will be considered in the calculations. After that, the result must show that the buoyancy force is bigger than the gravity force *Fb* > *Fg* so that the boat will be floating safely as shown in Figure 8.

### 3.2. Slider-Crank Mechanism

The main mechanism to open the gates is a Slider–Crank mechanism as shown in Figure 9, and it can be described as a mechanism of one degree of freedom, which consists of four rigid bodies connected to each other by three revolute joints and one prismatic joint to allow relative motion as illustrated in Figure 9. The four rigid bodies are illustrated as two links, one slider, and the ground (base) where they are connected to each other to allow linear motion.  Figure 10 shows the slider-crank displacement analysis; the graph of the slider-crank mechanism for displacement is matching the need very well. The theoretical results must be obtained by the experimental test.

### 3.3. Helical Gear Mesh

Using Ansys software, helical gears stresses will be designed to find the factor of safety. The yield stress of the grey cast iron is 130 MPa.  Figure 11 shows a primary result where the maximum stress is 62.33 MPa (the red color), while the blue is the lowest stress. Factor of safety =(130/62.335)=2.08 which is acceptable and safe as well.

RETRACTED

### 3.4. Water Pool Chemical Treatment

The following are many factors that need to be considered:

- Taking in consideration the size of the containers that will store the chlorine and pH acid.
- The time that it takes to release all chlorine and pH acid from the containers.
- The sensor design to give the red-light alarm when chlorine and pH acid are below the required level.
- The amount of chlorine and pH acid depends on the pool size.

Figure 12 below shows the process of the water pool treatment boat. The sensor will send a signal to the control logic when the chlorine and pH are below the required level. The control logic will display a red light in the remote control to tell the user that the swimming pool needs a chlorine and pH treatment. The user will release the chlorine and pH acid from the boat into the swimming pool by pushing a button from the remote control. After pushing the button, the red light will turn off and immediately will appear to the user to “move to the most far point,” so that the user will move the boat to the most far point of the swimming pool.

Since all the swimming pools use pumps to pump and circulate the water, the chlorine and pH will be circulated and spread in the swimming pool with time. After moving the boat into a different point of the swimming pool, which is far away from the release point. The sensor will start to check again the amount of the chlorine and pH acid after 15 or 20 minutes of the last release. A rectangular or square swimming pool was chosen that has a water volume of 40 cubic meters with two different amounts of depths as shown in Figure 13. We will take the swimming pool that has 40,000 litres of water as instance.

The amount needed per swimming pool size is provided in Table 1. The recommended size of the container is listed in Table 2.

Stabilised chlorine means cyanuric acid added to the chlorine to increase the time of the chlorine to remain in the swimming pool and not to evaporate quickly [2, 23–25]. Unstabilised is the opposite of the stabilised where the chlorine only will be used. The density of the chlorine acid is 2.994 *kg*/*m*^3^ at normal temperature and pressure is 20°C and 1 atm. In Table 2, all the chlorine is expressed in millilitres (ml) and it is known that 1 ml = 1 cm^3^.

The design of the boat is multi-combination systems of pools treatment as shown in Figure 14.

The container will have a pump inside it to pump the chlorine and pH acid by the nozzle marked 1 in the picture above. Also, there will be a sensor to check the chlorine level and pH acid marked number 2, and will be wire connected to the controller [26–28]. When the chlorine and pH blow the required level, the controller will send a signal to the user by flashing blue light marked 3 in the picture. The controller will be located at the centre of the boat with green color in the picture. To make the re-filling and checking the amount of the chlorine and pH acid easy for the user, I made an opening at the top of the container that is numbered 4 in the picture. Finally, I made a circuit that show and describe what I have said above in Figure 15.

RETRACTED

The circuit model has been run to show that all the design works good and in proper way. In Figure 16, the model has been run to check the result accuracy and how the system works.

Figure 16 shows the graph of frequency mode from the first step where the sensor checks the level until the last step where the chlorine will be released, when the sensor represented by the red line in the graph find out that level of the chlorine is low. When the frequency is low the red line will shift up little from its original position as it is pointed in Figure 6. Then, the sensor will send a signal to the controller to flash the blue LED represented by the yellow line in the graph. After that the user will push the button to turn on the pump to release the chlorine into the swimming pool, which is represented in blue line. When the pump starts, the light will turn off automatically [29, 30]. The blue line is only shift up and down same as the red line. The pump will run for 15 seconds, which is represented by the green line.

### 3.5. Process Sheet

The manufacturing process for each part of the boat is shown in Table 3. This sheet contains number of parts which has three digits, first one is the number of assembly and the second are a number of sub-assemblies, while the third digit is a number of the part at sub-assembly. Also, this sheet contains the material of the product and the quantity of each part. In addition, determining how many kinds and type of process will be used to product parts and the machine in number of operations. The process sheets are listed below.

Table 4 shows the net shaft which will be in the front of the boat and which will be going to in Aluminum. Two parts of this is needed to connect the net by the boat; turning process is considered by lathe machine with one operation.

The boat net is shown in Table 5. This will be in Polylastic acid (PLA) and one part is needed. Cutting process is considered and it can be done by saw machine, while the other process is drilling to make the hole and it can be done by drilling machine.

Table 6 shows the propeller, which is going to be made of Polymer and one propeller, is needed for the boat because it will be used for rudders. To make the propeller, CNC machine is needed because it is very complex, so starting by cutting operation is considered then using drilling to make the bore for the shaft.

RETRACTED

The sub-assembly part of the slider gates is shown in Table 7, which will be made of Polylastic acid (PLA) and two parts will be needed because one for chlorine and the other for acid. Three processes are: first is slot cutting by milling machine to make the internal gates with four operations. The second process is cutting to make the outer shape by saw machine. Third one is drilling to make the bore for the connecting rod.

Table 8 shows the sub-assembly of the slider base, which holds the gates. It will be made of polylastic acid (PLA) and two parts of it will be needed. This base will be machined by two processes: first is path cutting by using milling machine with only one operation. The second one is cutting, which will be by saw machine with one operation.

The rudder arm which controls the direction of the boat is illustrated in Table 9. It will be made of Aluminum and two parts will be needed. To make the rudder is performed in two processes, first is cutting to make the outer shape by saw machine with one operation, while the second process is drilling by drill press to make three holes.

The sub-assembly of the rudder, which is rudder joint, is shown in Table 10. It will be made of Aluminum and two parts will be needed of it. Three processes in machining, first is cutting with one operation. The second one is drilling to make six holes by drilling machine and it will be connected to rudder arms. Third process is slot cutting to make the internal cut by slot machine.

The steering rod, which connects the rudder to the motor, is shown in Table 11. It will be made of Aluminum and two parts of it are needed. Two processes in machining to make it, first is turning by lathe machine within one operation. The second process is bending with bar bending machine with two operations.

Table 12 shows the lifting pinion which transmits the power of the motor to control the net. It will be made of grey cast iron and two meshes of helical gear will be needed. Two processes needed to machine this pinion, first is tooth cutting by using milling machine. The second process is drilling for shaft bore by using drilling machine in one operation.

The slider rod shown in Table 13 will be made of Polylastic acid (PLA) and I need two parts of it. To manufacture this part, two processes will be needed; first one is cutting by using saw machine to make the outer shape with one operation. The second process is turning by using lathe machine in one operation.

RETRACTED

This is slider-crank rod, which connects the connecting rod to the gear-motor as shown in Table 14. It will be made by Polylastic acid (PLA) and two parts of it will be needed. Also, two processes will be used to machine this part; first one is cutting by lathe machine to make the outer shape. The second process is drilling the holes by using drilling press.

Table 15 shows the rudder pin which will connect the rudder arm by rudder joint. Two pieces of this will be needed to which will be made in Aluminum. It is very simple to manufacture it using turning process by lathe machine in one operation.

The worm gear shown in Table 16 transmits the power from motor to the lifting net. It will be made in grey cast iron and one mesh of it will be needed. It will be manufactured in three processes, first one is threading by CNC machine in one operation. The second process is drilling to make the bore of the gear. Third process is milling to make the pinion teeth in one operation.

The top cover of the boat shown in Table 17 is to keep the internal components safe from water. It will be made in transparent polymer and one part of it will be needed. It will be manufactured in one process, which is milling by CNC machine and three operations will be needed to make it done.

Finally, the gear-motors shown in Table 18 are to keep them safe from water. It will be made in transparent polymer and one part will be needed. It will be manufacturing by two processes, first one is milling by CNC machine and two operations will be needed to make it done. The second process is drilling to open three support holes.

## 4. Discussion

Furthermore, important tasks will be mentioned over systematically. The problem definition about swimming pool problems happening consistently has been reviewed. Likewise, swimming pool problems depend on source of it either way causing from human, climate, and environment conditions. In addition, to clear them out for the reader as referring before lookalike such as: chlorine reduction, pH decreases by time, and recreational water illnesses (RWIs). NAS offers smart and instantaneous security. The range of people that the boat could be very useful for is too wide; it can be a safety guard for children, and adults including the elderly. NAS is considered an environment friend as it has a relation with balancing chemical components in water of swimming pools, which has an impact on the air that people around it inhale. Filtering swimming pools water is killing a wide range of bacteria growing after swimming in the pool for a long time and they keep growing by the time unless there is something stopping them, which is the normal level of chlorine and acid in the water. In this way, the safety vibration sensor should be mentioned. It works by sensing the bandwidth of signals that come from wave conversation, which happens because of someone falling in the water.

RETRACTED

## 5. Conclusions

The vibration sensor offers perfection readings and exposes them into three ways of alerting. First, by showing a message in the LCD display of the remote. Second, by making sound through a whistle chip in the boat itself. Third, by making alarms by displaying lights on the boat as well, this will be much more obvious to see them in general! In addition, for reduction of chlorine or acid levels; there are two sliders containing medicine one for chlorine and the other one for acid. Both work when needed by human decision and condition in general. Each slider contains four rooms to keep medicine inside and ready to be dropped to do the expected object. In addition, calculations for mechanical components have been done, but some was done manually and the other by using several softwares such as Ansys, Analytix, and MitCalc on slider-crank, helical, and worm gears. After that, NAS has been designed and drawn using SolidWorks. Clearly, some analysis software has been used on the outcome results which are Ansys, Analytix, and MitCalc.

## Figures and Tables

**Figure 1:** Bacteria in swimming pools.

**Figure 2:** Patented on smart device for swimming pools.

**Figure 3:** Patented on smart flying boat.

**Figure 4:** Patented on motion sensor.

**Figure 5:** Speaker cords.

**Figure 6:** Raspberry Pi controls.

**Figure 7:** Overall view of the novel automated system.

**Figure 8:** Buoyancy force free body diagram.

**Figure 9:** Slider-crank mechanism free body diagram.

**Figure 10:** AC displacement against *θ*_2_.

**Figure 11:** Gear equivalent (von-mises) stress.

**Figure 12:** The process of the water pool.

**Figure 13:** The size of swimming pool treatment boat diagram.

**Figure 14:** An alternative design of swimming pool treatment boat diagram.

**Figure 15:** Control circuit.

**Figure 16:** The system identification.

**Table 1:** The amount needed per swimming pool size [22].

Pool volume litres	Stabilised pools daily dosage		Unstabilised pools daily dosage	
	Granular pool chlorine (g)	Liquid pool chlorine (ml)	Granular pool chlorine (g)	Liquid pool chlorine (ml)
10,000	50	200	80	400
20,000	100	400	160	800
30,000	150	600	240	1200
40,000	200	800	320	1600
50,000	250	1000	400	2000
60,000	300	1200	480	2400

**Table 2:** The size of the containers of swimming pool.

Model for each swimming pool in litres	The size of containers for stabilised pools (cm^3^)	The size of containers for unstabilised (cm^3^)
10,000	10*L* × 5*W* × 4*H*	12.5*L* × 6*W* × 5.5*H*
20,000	12.5*L* × 6*W* × 5.5*H*	13*L* × 9*W* × 7*H*

RETRACTED

**Table 3:** Process sheet of the bottom body of the boat.

Part No.	01.01.01		

Part name	Boat body		

Material	Aluminum		

No. of	1		

Process no.	Process name	Machine type	No. of operations

1	Cutting	Lathe machine	5

2	Drilling	Drill press	15

**Table 4:** Net shaft.

Part No.	01.02.01		

Part name	Net shaft		

Material	Aluminum		

No. of	2		

Process no.	Process name	Machine type	No. of operations

1	Turning	Lathe machine	1

**Table 5:** Net of the boat.

Part No.	01.02.03		

Part name	Boat net		

Material	Polylastic acid (PLA)		

No. of	1		

Process no.	Process name	Machine type	No. of operations

1	Cutting	Saw machine	1

2	Drilling	Drill machine	2

**Table 6:** Propeller.

Part no.	01.03.01		

Part name	Propeller		

Material	Polymer		

No. of	1		

Process no.	Process name	Machine type	No. of operations

1	Cutting	CNC machine	1

2	Drilling	CNC machine	1

**Table 7:** Slider gates.

Part No.	01.04.01		

Part name	Slider gates		

Material	Polylastic acid (PLA)		

No. of	2		

Process no.	Process name	Machine type	No. of operations

1	Slot cutting	Milling machine	4

2	Cutting	Saw machine	1

**Table 8:** Base of the slider.

Part No.	01.04.02		

Part name	Slider base		

Material	Polylastic acid (PLA)		

No. of	2		

Process no.	Process name	Machine type	No. of operations

1	Path cutting	Milling machine	1

2	Cutting	Saw machine	1

**Table 9:** Rudder arm.

Part No.	01.05.01		

Part name	Rudder arm		

Material	Aluminum		

No. of	2		

Process no.	Process name	Machine type	No. of operations

1	Cutting	Saw machine	1

2	Drilling	Drill machine	3

**Table 10:** Rudder joint.

Part No.	01.05.02		

Part name	Rudder joint		

Material	Aluminum		

No. of	2		

Process no.	Process name	Machine type	No. of operations

1	Cutting	Saw machine	1

2	Drilling	Drill machine	6

3	Slot cutting	Saw machine	1

**Table 11:** Steering rod.

Part no.	01.05.03		

Part name	Steering rod		

Material	Aluminum		

No. of	2		

Process no.	Process name	Machine type	No. of operations

1	Turning	Lathe machine	1

2	Bending	Bar bending machine	2

**Table 12:** Pinion.

Part No.	01.02.04		

Part name	Lifting pinion		

Material	Grey cast iron		

No. of	2		

Process no.	Process name	Machine type	No. of operations

1	Tooth cutting	Milling machine	1

2	Shaft hole	Drilling machine	1

**Table 13:** Slider rod.

Part No.	01.04.03		

Part name	Slider rod-1		

Material	Polylastic acid (PLA)		

No. of	2		

Process no.	Process name	Machine type	No. of operations

1	Cutting	Saw machine	1

2	Turning	Lathe machine	1

**Table 14:** Connecting slider rod.

Part No.	01.04.04		

Part name	Slider rod-2		

Material	Polylastic acid (PLA)		

No. of	2		

Process no.	Process name	Machine type	No. of operations

1	Cutting	Saw machine	1

2	Drilling	Press drilling	2

RETRACTED

**Table 15:** Rudder pin.

Part No.	01.05.04		

Part name	Rudder pin		

Material	Aluminum		

No. of	2		

Process no.	Process name	Machine type	No. of operations

1	Turning	Lathe machine	1

**Table 16:** Worm gear.

Part No.	01.02.05		

Part name	Worm gear		

Material	Grey cast iron		

No. of	2		

Process no.	Process name	Machine type	No. of operations

1	Threading	CNC machine	1

2	Drilling	CNC machine	1

3	Milling	CNC machine	1

**Table 17:** Cover of the boat.

Part No.	01.08.01		

Part name	Cover of the boat		

Material	Polymer		

No. of	1		

Process no.	Process name	Machine type	No. of operations

1	Milling	CNC machine	3

**Table 18:** Cover of motors.

Part No.	01.08.01		

Part name	Cover of the motors		

Material	Polymer		

No. of	1		

Process no.	Process name	Machine type	No. of operations

1	Milling	CNC machine	2

2	Drilling	CNC machine	3

## Data Availability

The data of this study will be available on reasonable request.
